# Porous materials of nitrogen doped graphene oxide@SnO_2_ electrode for capable supercapacitor application

**DOI:** 10.1038/s41598-019-48951-2

**Published:** 2019-09-02

**Authors:** Sivalingam Ramesh, H. M. Yadav, Young-Jun Lee, Gwang-Wook Hong, A. Kathalingam, Arumugam Sivasamy, Hyun-Seok Kim, Heung Soo Kim, Joo-Hyung Kim

**Affiliations:** 1 Department of Mechanical, Robotics and Energy Engineering, Dongguk University-Seoul, Pil-dong, Jung-gu, 04620 Seoul, Republic of Korea; 2 Department of Energy and Materials Engineering, Dongguk University-Seoul, Pildong-ro 1 gil, Jung-gu, Seoul, 04620 Seoul Republic of Korea; 3 Department of Mechanical Engineering, Inha University, Inha-ro 100, Nam-gu, Incheon, 402-751 Republic of Korea; 4 Millimeter-wave Innovation Technology (MINT) Research Center, Dongguk University-Seoul, Pil-dong, Jung-gu, 04620 Seoul, Republic of Korea; 5 Department of Chemical Engineering Area, Central Leather Research Institute (CLRI-CSIR), Adyar, Chennai 600020 India; 6 Division of Electronics and Electrical Engineering, Dongguk University-Seoul, Pil-dong, Jung-gu, 04620 Seoul, Republic of Korea

**Keywords:** Supercapacitors, Electrocatalysis

## Abstract

The porous materials of SnO_2_@NGO composite was synthesized by thermal reduction process at 550 °C in presence ammonia and urea as catalyst. In this process, the higher electrostatic attraction between the SnO_2_@NGO nanoparticles were anchored via thermal reduction reaction. These synthesized SnO_2_@ NGO composites were confirmed by Raman, XRD, XPS, HR-TEM, and EDX results. The SnO_2_ nanoparticles were anchored in the NGO composite in the controlled nanometer scale proved by FE-TEM and BET analysis. The SnO_2_@NGO composite was used to study the electrochemical properties of CV, GCD, and EIS analysis for supercapacitor application. The electrochemical properties of SnO_2_@NGO exhibited the specific capacitance (~378 F/g at a current density of 4 A/g) and increasing the cycle stability up to 5000 cycles. Therefore, the electrochemical results of SnO_2_@NGO composite could be promising for high-performance supercapacitor applications.

## Introduction

The nanotechnology of graphene-based materials are widely fabricated as active electrode for supercapacitor applications in presence of various strong electrolytes. In particular, the graphitic carbon electrodes are important role in the supercapacitor device applications^1–6^. Graphene is 2D carbon materials that contains high thermal conductivity, electrical conductivity, carrier mobility, and lateral quantum efficiencies. The carbon based materials are great interest because of the increasing the electronic capacity, mechanical properties, and superior chemical stability for photovoltaics, supercapacitors, and fuel cells applications^5,7–12^. The electrochemical performance of porous carbon material as electrical double layer capacitors (EDLC) is mainly depends on porosity, electrical conductivity, its dielectric constant, and various electrolytes. Based on the properties, the hybrid materials are classified into ultra-capacitor and conventional capacitors in the electrochemical reaction and its mechanism^13–17^. Recently, the N-doped graphene oxides (NGO) are widely used as electrode materials for supercapacitor, sensors and batteries studied in detail^18–20^. The NGO-metal oxides were synthesized to improve the electrochemical properties such as rate capability by using different catalyst^21,22^. Already the numerous research work reported on the NGO with metal oxides fabrication via CVD and thermal annealing process for supercapacitor and batteries applications. The various nanostructured metal oxides are fabricated in the electrochemical studies for increasing the specific capacitance and cyclic stability. In particular, the tin oxide (SnO_2_) is an n-type semiconducting material and its excellent chemical properties allow to fabricate electrodes, which used as the candidate for supercapacitor applications^23,24^. The nanostructured SnO_2_ is the most favorable metal oxides due to its increasing the capacitance, low cost, less poisonousness, and wide band gap ~3.6 eV. The various nanostructured SnO_2_/carbon composite was synthesized by hydrothermal process for electrochemical supercapacitor, sensors, and solar cells^25–29^. The SnO_2_ and RuO_2_ mixtures are used in the electrode materials for storage properties with an excellent cyclic stability^30^. The SnO_2_/graphene composite reported the increasing electrochemical performance and cyclic stability via microwave synthesis^31^. The construction of Ni/SnO_2_ composite shows an excellent capacitance and cyclic retention reported in the literature^32^. The hierarchical SnO_2_ composite displays the specific capacitance of ~188 F/g with 2000 cycles^33^. In the present study, SnO_2_@NGO composite was synthesized and it’s electrochemical properties investigated by CV analysis. The SnO_2_@NGO composite was analyzed by using Raman, XRD, XPS, BET, SEM, EDS, and HR-TEM analysis. Furthermore, the SnO_2_@NGO composite was studied by CV, GCD, and EIS techniques with 6 M KOH electrolyte.

## Results and Discussion

### Structural and surface morphology of SnO_2_@NGO

The schematic illustration of SnO_2_@NGO synthesis via thermal reduction process is depicted in Fig. 1. The Raman spectral analysis used to study the carbon-based materials and its defect structure. Figure 2(a) represent the Raman results of graphene oxide (GO) and NGO obtained by a thermal reduction reaction. The properties of graphene materials are represented at 1,580 cm^−1^ to the E_2g_ peaks of sp^2^ C atoms, and D band at 1,350 cm^−1^, which was ascribed to the breathing modes of the A_1g_ symmetry^34^. These peaks provide the information of local defects and disorder behavior of NGO by Raman spectroscopy (Fig. 2a). The Raman peaks represented that the D band at 1358 cm^−1^ and G bands 1597 cm^−1^ in the NGO structure. Moreover, the D/G intensity of NGO decreased when comparted to GO composite. The intensity change is may be due to the reduction of the NGO materials by thermal reduction process in the sp^2^ carbon structure. The peak position at lower wave numbers represent the different vibration modes of SnO_2_ nanoparticles in the NGO composite^35,36^.

**Figure 1:** Schematic illustration of SnO_2_@NGO synthesis via thermal reduction process.

**Figure 2:** (**a**) Raman, and (**b**) XRD of SnO_2_@NGO composite.

The XRD studies of GO indicated the peak at about 2θ = 10.80° with d -spacing 0.89 nm. The typical XRD peak of GO confirmed the well exfoliated carbon sheets in graphite structure has been reported previously^37–39^. The peak position at 2θ = (9.84° and 19.7°), corresponds to the (002) and (100) planes of GO materials. This may be due to the thermal reduction of GO to graphitic crystal structure in presence of high temperature. In addition, the diffraction pure SnO_2_ was studied in previous reports^40–43^ and SnO_2_@NGO diffraction peaks are represented in Fig. 2(b). The XRD of SnO_2_@NGO composite at 26.57°, 33.87°, 37.86°, 52.26°, 54.93°, 57.87°, 62.15°, 65.33°, and 71.28° are clearly distinguishable and corresponding planes (110), (101), (111), (211), (220), (002), (310), (301) and (202), respectively. The structure of tetragonal confirmed the PDF file no: JCPDS 41–1445. Therefore, the SnO_2_@NGO composite, which might be due to the exfoliation of NGO sheets at 550 °C by thermal reduction process.

Figure 3 represent the XPS peaks of SnO_2_@NGO composite. The survey spectrum (Fig. 3d) indicates that C 1s (285), O 1s (532), and Sn3d (487) eV, which complete the effective adornment of SnO_2_ nanoparticles onto the NGO surface. The Fig. 3c of Sn3d shows the main peaks of (3d_5/2_) and 3d_3/2_ corresponds to the binding energies of 487.0 eV and 495.5 eV, respectively. The binding energy difference between Sn3d_5/2_ and Sn3d_3/2_ almost ~8.7 eV. These results confirmed the identical to the binding energies of SnO_2_ and compared to the previous reports^44–46^.

**Figure 3:** XPS results of (**a**) C 1s (**b**) O 1s (**c**) Sn 3d and (**d**) survey spectrum of SnO_2_ @NGO composite.

Figures 4 and 5 represent morphological behaviors of SnO_2_@NGO composite studied by FE-TEM analysis. The (Fig. 4a–c) morphology of shows that altered the magnifications of NGO composite. The nanocrystalline SnO_2_ nanoparticles was decorated on the NGO and size of the particles in the range of ~10–20 nm (Fig. 4d). The high-resolution TEM of SnO_2_@NGO composite (Fig. 4a–c) represent the distance of the SnO_2_ nanoparticles are ~0.28 nm, matching to the (110) plane of SnO_2_. The SAED image of the SnO_2_@NGO (Fig. 4h) represent that the nanocrystalline behavior and this results consistent with XRD analysis of the composite. Figure 5 shows the different magnifications of SEM, SEM-EDS results confirms the C, O, N and Sn (Fig. 6) elements of the composite. In these results the N-doping level (32 wt %) on GO was achieved by simple hydrothermal method. The BET results are depicted in the Fig. 7. The surface area of the SnO_2_@NGO composite of about ~180 m^2^/g, pore volume of 0.27 cm^3^/g, and pore area of ~130 m^2^/g. The BJH analysis results are confirmed a mean pore size of the nanoparticles are ~(10–20) nm in the SnO_2_@NGO composite.

**Figure 4:** (**a**–**c**) TEM morphology of NGO materials, (**d**–**g**) HR- images of SnO_2_@NGO composite and (**h**) SAED pattern of composite.

**Figure 5:** (**a**–**f**) SEM-Morphology of SnO_2_@NGO composite.

**Figure 6:** (**a**–**b**) SEM-EDS and (**c**) C 1s (**d**) O 1s (**e**) N 1s and (**f**) Sn 3d morphology of SnO_2_@NGO composite.

**Figure 7:** BET results of (**a**–**d**) SnO_2_@NGO composite.

### Electrochemical measurements of SnO_2_@NGO composite

The electrochemical results of GO, RGO, NGO and SnO_2_ composite and its supercapacitor properties were reported in the previous studies^26,47–49^. The SnO_2_@NGO composite was studied by cyclic voltammetric analysis results are shown in Fig. 8 and Table 1. The composite results indicate the ideal capacitive nature showing the rectangular profile owing to outstanding trend for supercapacitor. The trend of CV curves of composite electrodes, rectangular properties and corresponding increase of current than that of pristine SnO_2_. These properties of composite shows the increasing the specific capacitance because of the combined influence from EDLC and pseudo capacitance of the composite. Figure 8a represent the CV results of SnO_2_@NGO composite electrodes with the scanning rate from (10–100) mV s^−1^ in presence of 6 M KOH aqueous electrolyte. The electrochemical properties were studied the potentials range between (−0.2 and 0.8 V), it can be seen that the increasing the capacitance behaviors between the electrode and electrolyte. The scan rates increases, the current density also increases, because of the anodic and cathodic current change towards the reversible reaction. This fast redox or reversible reactions occurring between the electro-active material/electrolyte interfaces in presence 6 M KOH. Because of the CV represent a slight alteration with certain number of functional groups react in the NGO and SnO_2_ nanoparticles. The specific capacitance of SnO_2_@NGO electrodes are intended from the CV curves. The cyclic voltammetry results are shown Fig. 8a. In this CV experiments, the scan rate increased from 10 to 100 mV s^−1^ and also increases the electrochemical supercapacitor properties. The enhancement of electrochemical properties of the composite is mainly denoted to the more electroactive sites via EDLC and pseudo capacitance arises in the SnO_2_@NGO composite. Further, the SnO_2_ nanoparticles at the NGO matrix successfully decorated and low internal resistance with high electrical conductivity of the composite for electrochemical reversible reaction^26,47–49^.

**Figure 8:** (**a**) CVs of the SnO_2_@NGO composite electrodes at various scan rates of (10–100) mV s^−1^ in 6 M KOH. (**b**) Charge/discharge profiles of the composite electrode at different current densities (4, 8.5, and 12.6) A/g. (**c**) Variation of specific capacitance as a function of cyclic number at a current density of 4.0 A/g, (**d**) EIS, and (**e**) the effect of Energy density *vs*. Power density.

**Table 1:** Parameters for the supercapacitor of SnO_2_ and SnO_2_@NGO electrodes reported in the literature.

Electrode material	Preparation method	Capacitance (F/g)	Cyclic stability	Ref.
SnO_2_@C nanoparticles	Calcination process at (500–700) °C	37.8 F/g at 5 mV/s	NA	^54^
SO4^2−^/SnO_2_ nanocomposite	Alkaline hydrolysis	51.95 F/g at 5 mV/s	7.5% loss after 2,000 cycles	^55^
Hydrous SnO_2_ Thin films composite	Chemical Synthesis of Thin film	25 F/g at 5 mV/s	NA	^56^
MWCNT/SnO_2_ composite	Decoration by sonochemical process	133.33 F/g at 0.5 mV/s	10% loss after 500 cycles	^57^
GO/SnO_2_	Spray pyrolysis	61.7 F/g at 1 A/g	1% loss after 106 cycles	^52^
SnO_2_/Graphene	Microwave assisted one-pot reaction	99.7 F/g at 5 mV/s1	NA	^48^
GNs/SnO_2_–MWCNTs	Chemical method followed by calcination	224 F/g at 10 mA	8% loss after 6000 cycles	^58^
RGO/SnO_2_ composite	Microwave assisted deposition	348 F/g at 50 m A g^−1^	2% loss after 1,000 cycles	^59^
**SnO**_**2**_ **@NGO** **composite**	**Thermal reduction** **process**	**378** **F**/**g** **at 4** **A**/**g**	**11% loss after** **5**,**000 cycles**	**This work**

NA-Not available.

Furthermore, the SnO_2_@NGO composite for charge-discharge test from the GCD curves represented in Fig. 8(b). The GCD curves of composite electrodes are increases the current density of 4, 8.5 and 12.6 A/g by using 6 M KOH solution. The GCD results evidently designates the triangular shape of the composite materials and the contribution of EDLC and pseudo capacitance properties from CV analysis. The composite electrodes are confirmed the higher discharge time than that of pristine SnO_2_ composite represent the increasing specific capacitance with stronger electrolytes^26,47–49^.

The specific capacitance values are ~378 F/g, 345 F/g, and 230 F/g at the current density of 4, 8.5, and 12.6 A/g, respectively. The Fig. (8c,d) represent the cyclic retention and corresponds to the current density (*vs*) its specific capacitance values. The trend of the specific capacitance values was decreased, as the current density increased 4, 8.5, and 12.6 A/g. Because of the diffusion of the electrolyte ions, depends on the morphology, surface of the materials and concentration of the SnO_2_ and NGO components. The electrochemical properties of the SnO_2_@NGO nanoparticles was compared to the previous reports for supercapacitor applications^50–52^.

In addition, the SnO_2_@NGO composite, energy density and power density results are shown in Fig. 8(e,f). The cyclic stability is the important property of the electrode for practical applications in the supercapacitors. Figure 8(c) shows the GCD analysis at a current density of 4 A/g for 5,000 cycles. After 2,000 cycles, the composite electrode maintained 89% of its original performance, which signifies of electroactive material has better cyclic stability^49,53^ and reversibility of the GCD process.

Furthermore, the EIS results were estimated at open circuit potential by relating the various ac voltages in the frequency range from 0.1 Hz to 100 kHz. Figure 8(d) represent the EIS result of Nyquist plots for SnO_2_@NGO composite, which is indicate that the real and imaginary parts of EIS results, respectively. First, the smaller semi-circular loop at higher frequencies is attributed to the Faradaic reactions in presence of the 6 M KOH electrolyte. The lower frequency region of the EIS increases due to the capacitive nature of SnO_2_@NGO composite. The phase angle of EIS of composite electrode was perceived to be higher than 45° and low frequencies demonstrating the electrochemical capacitive nature of the composite materials. In this regard, the charge transfer resistance (Rct) of the NGO and composite electrodes are ~36 and 38, respectively. In this lower value of Rct represent the stable electrochemical performance. The low-frequency region of the impedance analysis results are called Warburg resistance of diffusion behavior in presence of 6 M KOH with in the electrodes. The vertical slope of Warburg curves specifies the rapid development of an electric double-layer in the composite because of quick ion diffusion in presence of 6 M KOH electrolyte for supercapacitor applications^49,54^.

## Conclusions

The porous material of SnO_2_@NGO composite synthesized by thermal reduction process and studied their electrochemical characteristics towards high-performance supercapacitors. The Raman, X-ray diffraction, and photoelectron spectroscopy analysis reveals the successful formation of SnO_2_@NGO composite. The specific capacitance of the SnO_2_@NGO composite displayed the capacitance ~378 F/g at a current density of 4 A/g in the 6 M KOH solution. Moreover, the composite electrode exhibited an excellent cycling stability at 4 A/g. The composite electrode maintained 89% of its original performance after 5000 cycles in presence of 6 M KOH electrolyte, there by representing the plausible applicability for energy storage applications.

## Materials and Methods

### Materials

The graphene oxide from graphite flakes, sulfuric acid (H_2_SO_4_,), phosphoric acid (H_3_PO_4_), potassium permanganate (KMnO_4_), potassium hydroxide (KOH), hydrogen peroxide (H_2_O_2_, 30%) in this experiment. The tin (IV) chloride pentahydrate (SnCl_4_.5H_2_O, 98%), ammonia solution (NH_3_, 30%), N-methyl-2-pyrrolidone and polytetrafluorethylene (PTFE) were chemicals received from Sigma-Aldrich, South Korea.

### Graphene oxide synthesis (GO)

The graphene oxide (GO) materials were developed by Hummer’s technique in the previous reports^27–29^. The graphite (5 g), H_2_SO_4_ (400 mL), H_3_PO_4_ (50 mL), and KMnO_4_ (18 g) were mixed in the three-neck flask using a magnetic stirrer at 40 °C and continually stirred for 48 h to achieve the complete conversion from graphite. After that, the reaction mixture was changes from dark purple to greenish brown color and the calculate amount 20 mL of H_2_O_2_ was added to complete the conversion of GO. The GO was purified by using 1 M of HCl or ethanol and then purified the oven at 80 °C for 12 h.

### N-Doped graphene oxide synthesis (NGO)

The calculated amount of 0.5 g of GO was distributed in the 300 mL of distilled water followed by ultra-sonication and the solution becomes the brownish GO suspension. The GO suspension and required amount of 20 mL of excess of water is added and stirred for 4 h and filtered/dried in the vacuum oven at 90 °C for 4 h. Then the calculated amount of 1 g of urea and ammonia and excess of 20 mL of ammonia was added and continuously stirred at 90 °C for 12 h. Finally, the GO product was dried in the oven at 200 °C for 12 h, and purified by using ethanol solvent.

### SnO_2_@NGO composite synthesis

Briefly, 0.2 g of GO was distributed in 150 mL of water and sonication for 1 h to become the homogeneous solution. Then the calculated amount of 1.2 g of stannous chloride, 25% of 10 mL ammonia solution was added to the GO solution to maintain the basic medium. Afterwards, the reaction GO solution was refluxed at 200 °C for 8 h by using three neck flask with condenser. Then, the reaction becomes changed to black color product of SnO_2_@NGO and dried in the vacuum oven at 180 °C for 12 h. Further, the SnO_2_@NGO sample was calcination at 550 °C for 8 h and collected the product for further characterization.

### Preparation of electrochemical analysis

The CV experiment was studied in the regular three-electrode system connected through Autolab PGSTAT302N (Metrohm, Netherlands). The SnO_2_@NGO composite (working electrode), carbon black, and PVDF in the stoichiometric of 75: 15: 10 and dispersed in the n-methyl 2-pyrrolidone. The resulted black paste was then covered onto a nickel wire collector and dried at 110 °C for 12 h. The mass loading of the SnO_2_@NGO composite is around 1.5 mg cm^−2^. In this experiment, platinum wire (counter electrode) and Ag/AgCl (reference electrode) were fabricated in the CV analysis. The synthesized SnO_2_@NGO composite and its electrochemical properties were determined by cyclic voltammetry analysis. The CV curves were documented at various scan rates (10, 20, 40, 60, 80, and 100) mV s^−1^ in a potential range of (−0.2 to 0.8) V. The GCD curves were acquired at various current densities (4, 8.5 and 12.6) A/g and EIS results in the frequency range of (0.1 Hz to 100 kHz). The capacitance of SnO_2_@NGO composite was designed from the CV Eq. (1), and GCD curves Eq. (2) were shown in the previous reports^30–33^.

### Materials characterization

Raman studies were analyzed in the range (100 to 4000 cm^−1^) by using RM200 confocal Raman spectroscopy. The composite was studied the wide-angle XRD analysis documented by Rigaku Rotaflex (RU-200B) diffractometry in presence Cu Kα radiation. The morphological properties of SnO_2_@NGO were analyzed by using FE-SEM-4800, and JEM-2010F FE-TEM, Hitachi Japan. The SnO_2_@NGO composite was examined by X-ray photoelectron spectroscopy by (Thermal Fisher Scientific, USA) with Kα radiation.
